# Sentinel Node Mapping in Ovarian Tumors: A Study Using Lymphoscintigraphy and SPECT/CT

**DOI:** 10.1155/2024/5453692

**Published:** 2024-02-23

**Authors:** Saeideh Ataei Nakhaei, Ramin Sadeghi, Sayyed Mostafa Mostafavi, Giorgio Treglia, Malihe Hassanzadeh, Maryam Esmaeilpour, Negar Sadat Taheri, Marjaneh Farazestanian

**Affiliations:** ^1^Nuclear Medicine Research Center, School of Medicine, Mashhad University of Medical Sciences, Mashhad, Iran; ^2^Department of Computer Engineering, University of Isfahan, Isfahan, Iran; ^3^Imaging Institute of Southern Switzerland, Ente Ospedaliero Cantonale, Bellinzona, Switzerland; ^4^Faculty of Biomedical Sciences, Università della Svizzera Italiana, Lugano, Switzerland; ^5^Faculty of Biology and Medicine, University of Lausanne, Lausanne, Switzerland; ^6^Women's Health Research Center, Mashhad University of Medical Sciences, Mashhad, Iran

## Abstract

**Purpose:**

Ovarian cancer in the early stage requires a complete surgical staging, including radical lymphadenectomy, implying subsequent risk of morbidity and complications. Sentinel lymph node (SLN) mapping is a procedure that attempts to reduce radical lymphadenectomy-related complications and morbidities. Our study evaluates the feasibility of SLN mapping in patients with ovarian tumors by the use of intraoperative Technetium-99m-Phytate (Tc-99m-Phytate) and postoperative lymphoscintigraphy using tomographic (single-photon emission computed tomography/computed tomography (SPECT/CT)) acquisition.

**Materials and Methods:**

Thirty-two patients with ovarian mass participated in this study. Intraoperative injection of the radiopharmaceutical was performed just after laparotomy and before the removal of tumor in utero-ovarian and suspensory ligaments of the ovary just beneath the peritoneum. Subsequently, pelvic and para-aortic lymphadenectomy was performed for malignant masses, and the presence of tumor in the lymph nodes was assessed through histopathological examination. Conversely, lymphadenectomy was not performed in patients with benign lesions or borderline ovarian tumors. Lymphoscintigraphy was performed within 24 hr using tomographic acquisition (SPECT/CT) of the abdomen and pelvis.

**Results:**

Final pathological examination showed 19 patients with benign pathology, 5 with borderline tumors, and 6 with malignant ovarian tumors. SPECT/CT identified SLNs in para-aortic-only areas in 6 (20%), pelvic/para-aortic areas in 14 (47%), and pelvic-only areas in 7 (23%) cases. Notably, additional unusual SLN locations were revealed in perirenal, intergluteal, and posterior to psoas muscle regions in three patients. We were not able to calculate the false negative rate due to the absence of patients with involved lymph nodes.

**Conclusion:**

SLN mapping using intraoperative injection of radiotracers is safe and feasible. Larger studies with more malignant cases are needed to better evaluate the sensitivity of this method for lymphatic staging of ovarian malignancies.

## 1. Introduction

Ovarian cancer is diagnosed in the early stages of the disease in a significant proportion of cases [1]. Bilateral pelvic and para-aortic lymphadenectomy is recommended by FIGO (The International Federation of Gynecology and Obstetrics) in the early stage of ovarian cancer [2]. However, patients with total lymphadenectomy may suffer from complications such as blood loss, chronic lower limb lymphedema, lymphoceles, etc [3–5]. Furthermore, only a minority of these patients have lymph nodal involvement, and this information is crucial for the real benefit of routine lymph node dissection [6].

However, lymph nodal metastases upstage the disease [7], and in order to reduce the procedure-related morbidity of routine total lymph node dissection, sentinel lymph nodal (SLN) mapping in ovarian mass has been evaluated in the research setting over the past decade.

The aim of the present study is to assess the feasibility of ovarian SLN mapping using lymphoscintigraphy and tomographic acquisition (single-photon emission computed tomography/computed tomography (SPECT/CT)).

## 2. Materials and Methods

The study design was prospective. A total of 32 patients were diagnosed with an adnexal mass suggestive of a malignant ovarian tumor who included increased tumor marker (CA-125; cancer antigen 125) and sonographic characteristics confined to O-RADS (The Ovarian-Adnexal Reporting and Data System) 4 and 5 [8], during a period from May 2019 to Dec 2021, were eligible for inclusion in the study (Figure 1). All patients provided fully informed consent to the study before their enrollment. The study protocol was approved by the Local Ethics Committee of our institute (approval number: 931331).

Exclusion criteria were as follows: known advanced stage (FIGO stage II or greater) ovarian cancers; previous ovarian surgery; previous vascular surgery, lymphadenectomy, or lymph node sampling on the abdominal or pelvic region; history of lymphoma or malignant tumor in the abdominal or pelvic region; pregnancy or lactation.

After the opening of the abdomen and before the removal of the ovarian mass, two injections included standard doses of 18.5 MBq or 0.5 mCi/0.2–0.5 mL/each injection of Tc-99m-Phytate were performed in the proper ovarian ligament and the suspensory ligament, close to the diseased ovary and just underneath the peritoneum. Regarding the dose of the tracer, many studies (including several studies of our group) reported the feasibility of a 2-day protocol by 1 mCi total tracer with excellent results in breast cancer [9, 10]. In addition, in the previous study of our group, we also used the same low dose for ovarian tumors with excellent results of imaging the day after injection [11]. After a 15–20-min interval, to provide sufficient time for the lymphatic flow of the radiotracer, the adnexal mass was removed and sent for pathological (frozen-section) analysis. Subsequently, if a benign lesion or borderline ovarian tumor was revealed on the frozen section, lymph node dissection was not performed. However, SLNs identified transperitoneal using a handheld cesium iodide scintillation gamma probe (Surgiguide, Partonegar Persia) by searching the para-aortic and pelvic areas, and the locations of any detected SLNs were recorded. The criteria of SLN identification was a “hot” node with more than a 10-fold count as compared to the background. The background was measured from the thighs of the patients using gamma-probe. If a malignant ovarian tumor was found, the retroperitoneal space was opened, and SLNs were localized with the gamma-probe and assessed through histopathological analysis using hematoxylin and eosin staining. After the removal of the SLNs, the presence of radioactivity in the location from which they were removed was assessed, and no further action was taken if the radioactivity was ≤10% of the background. Subsequently, a complete standard staging procedure, including pelvic and para-aortic lymphadenectomy, was performed. The surgeon also recorded the location of non-SLNs removed. The histopathology of SLNs and non-SLNs was performed separately. The morning after surgery, all patients depending on the condition and mobility of the patient, were sent to the nuclear medicine ward for lymphoscintigraphy, including tomographic (SPECT/CT) acquisition of the abdomen and pelvis. Static images (10 min/image) in anterior and posterior views of the abdomen and pelvis were performed, followed by tomographic SPECT/CT images of the same regions using a SPECT/CT tomograph (Precedence SPECT/6-slice CT scanner; GE), equipped with dual 1.6-cm g-detectors and low-energy general-purpose collimators. Abdominal and pelvic SPECT data were obtained through a circular orbit, a 128 × 128 matrix, and six view angles over a total angle range of 360 and 25 s per stop, then CT scanning was performed (120 keV, 80 mAs, 3.75 mm-thick slices). Scintigraphic and SPECT/CT image interpretation was performed by two nuclear medicine physicians familiar with SLN mapping. The results of the lymphoscintigraphy were correlated with the intraoperative findings.

## 3. Results

Thirty-two patients were included in the study. The SLN mapping procedure was completed in 30 of 32 patients (94%).  Table 1 shows the characteristics of patients. In two patients with an endometrioma cyst, radiotracer injection was not performed due to the presence of adhesions, which prevented the access to the ovarian ligaments. The radiotracer was injected 13 times on the left side, 9 times on the right side, and 8 times bilaterally. The final pathological examination results showed 19 patients with benign disease, 5 with a borderline ovarian tumor, and 6 with a malignant ovarian tumor. The results of the frozen section analyses were confirmed at the final histopathological examination.  Figure 2 shows the hotspot locations identified with the gamma-probe and with SPECT/CT postoperatively. At least one SLN could be identified by gamma probing in all but three patients, thus resulting in a 90% detection rate. Moreover, postoperative SPECT/CT lymphoscintigraphy did not reveal any SLN in these three patients. Patients with malignant pathology all had at least one SLN harvested during surgery (100% detection rate). In four patients (Patients 3, 5, 7, and 26), postoperative SPECT/CT detected two hotspots on the same location of SLNs by gamma probing. SPECT/CT lymphoscintigraphy shows three aberrant locations for SLNs, including intergluteal, perirenal regions, and posterior to psoas muscle in Patients 4, 6, and 29, respectively (Figure 3). Overall, SLNs were identified in para-aortic/aortocaval areas in 6 patients (20%), pelvic/para-aortic areas in 14 (47%) patients, and pelvic-only areas in 7 (23%) patients in whom SLNs were detected. Most patients had ipsilateral lymphatic drainage to the ovarian injection side. Nevertheless, in this study, three patients (2, 24, and 29) had contralateral lymphatic drainage. In addition, in Patient 4, bilateral lymphatic drainage was observed. In the patients with bilateral ovarian injection (eight cases), lymphatic drainage was noticed on the right pelvic side/aortocaval region in two cases (Patients 3 and 15), left pelvic side/para-aortic region in two cases (Patients 18 and 23), bilateral pelvic side in two cases (Patients 6 and 13) and no SLNs in two cases. In 16 patients with para-aortic SLNs, injection sides were bilateral in 2 cases, the left side in 10 cases and the right side in 4 cases. In patients with malignant pathology, none had SLN or non-SLN involvement by histopathological examination. Adverse reactions to radiotracer did not occur in any of the patients during the 7-day follow-up period.  Figure 4 shows SPECT/CT lymphoscintigraphy images of Patient 24.

## 4. Discussion

The significance of ovarian SLN mapping in early ovarian cancer has been outlined in the literature. This is primarily due to two facts. First, Lago et al. [7, 12] and Uccella et al. [13] reported upstaging of early ovarian cancer by detected lymph node metastases. Second, systemic lymphadenectomy for nodal staging is accompanied by the risk of complications [5, 14]. In line with the studies already performed on ovarian SLN mapping, our study illustrates that SLN mapping of ovarian masses is feasible, resulting in a detection rate of 90% by using an intraoperative gamma probe. We summarized the information about the published studies on ovarian SLN mapping in addition to the current one (Table 2). In the majority of published studies, the radiotracer injection was performed with the adnexa still in situ. However, some studies [12, 22, 23] performed the radiotracer injection in the infundibulo-pelvic and utero-ovarian ligament stumps after the removal of the ovarian tumor, during the same or a subsequent surgical procedure. SLN detection rates ranged from 100% [12, 22] to 27% [23]. As such, more studies are needed to better explore the impact of tracer injection in ovarian SLN mapping. Notably, near-infrared fluorescent technology is unfortunately not available in all centers for the detection of ICG (indocyanine green)-stained SLNs. In addition, allergic reactions are reported to blue dyes during SLN mapping. Furthermore, SLN mapping using blue dye seems to be more affected with high body mass index [21]. As such, Tc99m-radiocolloids seem to be the preferred tracers for ovarian SLN mapping. Most of the studies that utilized Tc99m-radiocolloids as mapping material used a median dose of 37–74 MBq, which equals 1–2 mCi per injection. We used a low dose of Tc99m-Phytate (18.5 MBq equals 0.5 mCi per injection) with a relatively high SLN detection rate, which exposes the patients to a small amount of radiation. Considering the literature, we noted that injection just underneath the peritoneum resulted in a higher detection rate compared to ovarian cortex injection. As such, in line with most of the studies, we also performed the radiotracer injection in the suspensory and the infundibulo-pelvic ligaments with high success and detection rate. Previous studies used a median 15-min interval between Tc99m-radiocolloid injection and lymph node mapping, which seems enough to allow the flow of the radiotracer to the SLNs and cause an acceptable SLNs detection rate. In the current study, we used a waiting time of 15–20 min after injection with a comparable detection rate. Thus far, only three studies [11, 15, 20] on ovarian SLN mapping used imaging of SLNs using lymphoscintigraphy post-operatively rather than intraoperative count of the para-aortic or pelvic areas as the preferred method for SLN detection. In patients with benign disease who did not undergo lymph node dissection, this is the only method to show the exact location of SLNs. Adding SPECT/CT to the lymphoscintigraphy imaging ratifies this with a higher accuracy. To the best of our knowledge, except our study, only Speth et al. [20] already studied ovarian SLN mapping by postoperative SPECT/CT. Our study shows that hot spots were found isolated in the para-aortic and paracaval regions in 20%, in the pelvic region only in 23%, and in both the para-aortic/paracaval and the pelvic regions in 47% of the patients. In all but four patients, the SLNs were ipsilateral to the injection site. Among these four patients, three cases had contralateral lymphatic drainage and one patient was bilateral. These results are fairly similar to the previous studies in this regard [16–19, 21]. In some patients, postoperative SPECT/CT showed additional SLNs at the same location compared to only one SLN detected by gamma probing. This is because SPECT/CT has a better spatial resolution, and in particular, a significant body of evidence in the literature clearly shows that hybrid imaging increases the accuracy of scintigraphic studies in SLN mapping by providing a precise anatomical/functional correlation [24, 25]. In addition, SPECT/CT techniques and algorithms such as whole-body SPECT/CT (to discover aberrant sentinel nodes outside the conventional lymphadenectomy locations) and resolution recovery algorithms (to improve sentinel node detections via better resolution) would be helpful in the future studies. Moreover, SPECT/CT detects aberrant SLNs (e.g., intergluteal, perirenal) in unexpected locations, which are conventionally overlooked by intraoperative gamma probing. Specifically, these aberrant locations are important in the malignant ovarian mass where metastatic involvement of lymph nodes can be missed by routine intraoperative gamma probing. Moreover, the results of this study indicate that lymphatic drainage of the unilateral ovarian mass may be contralateral or bilateral. As such, it is important that bilateral lymph node locations are searched for SLN by intraoperative gamma probing. In addition to the detection rate in ovarian SLN mapping studies, false negative rate (and following sensitivity) is also an important index of the SLN mapping studies. However, a major limitation is the fact that because ovarian cancers are often diagnosed at an advanced stage of the disease, only a small group of patients with early ovarian cancer were considered in this study. On the other hand, definitive diagnosis of the type of adnexal mass (benign vs. malignant) prior to resection and frozen section is not possible, while the SLN mapping procedure should be performed before ovarian mass resection. As such, most of the studies did not include enough malignant ovarian mass cases for lymph node dissection and histopathological assessment, resulting in insufficient data to calculate false negative rate and sensitivity. In our study, no patients had involved lymph nodes and, as such, we were not able to calculate the false negative rate. To date, only five studies [11–13, 17, 21] had sufficient data to assess the sensitivity of SLN mapping in the lymphatic staging of ovarian tumors. SLN mapping and biopsy in ovarian tumors is actually in its infancy, and the feasibility of lymphatic mapping for ovarian masses is still under debate. Our study clearly showed that lymphatic mapping is feasible in ovarian masses using SPECT/CT as an adjunct. As malignancy of ovarian masses cannot be determined before surgery with certainty, benign or intermediate tumors would be invariably included in all studies in this topic, which limits the number of patients with pathologically involved regional lymph nodes (very few studies reported these cases thus far). Therefore, more studies with larger sample sizes are warranted to confirm the results of these studies. In agreement with several previous studies [26–28], the radiation safety of ovarian SLN mapping was also reiterated in our study.

## 5. Conclusion

SLN mapping is feasible in ovarian masses with a high detection rate confirmed by postinjection lymphoscintigraphy SPECT/CT and expected lymphatic drainage to pelvic and para-aortic areas. Harvesting SLNs in malignant ovarian masses is also possible. Larger studies with more malignant cases are needed for better evaluation of false negative rate and sensitivity.

## Figures and Tables

**Figure 1:** Flowchart of the patient's selection.

**Figure 2:** Location of hot spots found using intraoperative gamma probing. The hexagons are locations of hot spots found in patients (*n* = 9) with tumor on the right side. The circles are locations of hot spots found in patients (*n* = 13) with tumor on the left side. The squares are locations of hot spots found in patients (*n* = 8) with tumor on bilateral sides.

**Figure 3:** Aberrant ovarian sentinel lymph nodes (SLN) in the sagittal and transverse SPECT/CT lymphoscintigraphy. (a) and (b): intergluteal SLN; (c) and (d): peri-renal SLN; and (e) and (f): psoas region SLN.

**Figure 4:** Planar lymphoscintigraphy in the (a) anterior and (b) posterior views show hotspots in the mid-abdomen and left pelvic side. SPECT/CT shows the exact location of these hotspots compatible with para-aortic and left internal iliac sentinel lymph nodes in the (c, d) transverse and (e, f) coronal views.

**Table 1:** Characteristics of the patients (*N* = 30).

Patient number	Age (years)	CA125 (U/ml)	O-RADS/Max diameter of adnexal mass (cm) on ultrasonography	Injection side	Final pathology result	SLNs location on postoperative SPECT/CT lymphoscintigraphy (number of SLNs)	SLNs/non-SLN histopathological involvement
1	61	127	O-RADS 4/10	Left	Mucinous adenocarcinoma	Para-aortic (only on the gamma probing)	–/–
2	70	87	O-RADS 5/20	Right	Borderline serous cystadenoma	Para-aortic/left common iliac	—
3	46	51	O-RADS 4/15	Bilateral	Mature teratoma	Aortocaval (2)/right internal iliac	—
4	45	90	O-RADS 4/15	Right	Serous cystadenoma	Aortocaval/para-aortic/left and right internal iliac/left intergluteal region	—
5	41	45	O-RADS 4/15	Left	Benign epithelial tumor with ovarian torsion	Para-aortic (2)	—
6	56	75	O-RADS 5/20	Bilateral	Borderline serous cystadenoma	Right common iliac/left external and internal iliac/left perirenal (2)	—
7	25	42	O-RADS 4/15	Left	Benign epithelial tumor with ovarian torsion	Para-aortic (2)/left internal iliac	—
8	55	40	O-RADS 4/10	Bilateral	Serous cystadenoma	None	—
9	47	189	O-RADS 4/12.5	Bilateral	Endometrioma	None	—
10	55	0.1	O-RADS 4/15	Right	Serous cystadenoma	Aortocaval/right common iliac	—
11	50	28	O-RADS 4/20	Left	Serous cystadenoma	Aortocaval/left internal iliac	—
12	63	15	O-RADS 4/16	Right	Serous cystadenoma	Right common iliac	—
13	27	54	O-RADS 4/22	Bilateral	Mixed serous and mucinous cystadenoma	Para-aortic/right and left external iliac	—
14	40	35	O-RADS 4/22	Left	Serous cystadenoma	Left common iliac	—
15	63	144	O-RADS 5/8	Bilateral	Endometrioma	Right internal iliac	—
16	37	123	O-RADS 5/7	Right	Papillary serous cyst adenocarcinoma	Para-aortic/right common iliac (only on the gamma probing)	–/–
17	15	11	O-RADS 4/10	Right	Mature teratoma	None	—
18	41	23	O-RADS 5/11	Bilateral	Borderline mucinous cystadenoma (left) and endometrioma (right)	Left common iliac/left external iliac	—
19	34	38	O-RADS 4/8	Left	Mucinous cystadenoma	Left external iliac	—
20	49	28	O-RADS 4/9	Left	Mucinous cystadenoma	Para-aortic	—
21	63	10	O-RADS 4/15	Left	Fibrothecoma	Para-aortic	—
22	52	51	O-RADS 5/10	Left	Mature teratoma	Para-aortic/left external and internal iliac	—
23	84	18	O-RADS 5/12	Bilateral	Sex cord-stromal tumor	Para-aortic (only on the gamma probing)	–/–
24	38	361	O-RADS 4/7.7	Right	Papillary serous cyst adenocarcinoma	Para-aortic/left external iliac (only on the gamma probing)	–/–
25	18	210	O-RADS 5/24	Right	Germ cell tumor	Para-aortic/Right external iliac (only on the gamma probing)	–/–
26	49	435	O-RADS 4/17	Right	Borderline serous cystadenoma	Right internal iliac (2)	—
27	22	27	O-RADS 4/30	Left	Mucinous cystadenoma	Para-aortic	—
28	34	38	O-RADS 5/15	Left	Borderline serous cystadenoma	Para-aortic/left internal iliac	—
29	58	69	O-RADS 4/15	Left	Fibro-thecoma	Para-aortic/left external iliac/posterior to right psoas muscle region	—
30	50	230	O-RADS 5/13	Left	Malignant epithelial ovarian tumor	Para-aortic/left external iliac (only on the gamma probing)	–/–

**Table 2:** The published studies on ovarian sentinel node mapping.

First author/year	Study population/number of patients	Mapping material	Site of injection	Wait time after injection	SLNs location	Detection rate/false negative rate
Vanneuville/1991 [15]	Ablation of benign ovarian cyst or for tubal ligation/14	Tc-99m + rhenium sulfide colloid	Mesovarium (of normal ovaries)	4–6 hr scintigraphy	Aortic only 33%/both aortic and pelvic 67%	85.7%/NA
Negishi/2004 [16]	Ten endometrial cancer, one fallopian tube tumor/11	CH40 (charcoal solution)	Ovarian cortex	10 min	Aortic only 64%/ both aortic and pelvic 36%	100%/NA
Kleppe/2014 [17]	Patients with a pelvic mass suggestive of a malignant ovarian tumor/21	Tc-99m—albumin nanocolloid + blue dye	Proper ovarian and suspensory ligament	Minimum 15 min	Aortic only 67%/ pelvic only 9.5%/ both aortic and pelvic 24%	100%/0%
Hassanzadeh/2016 [11]	Patients with ovarian mass (cancer = 13,benign = 1, borderline = 21 patients)/35	Tc-99m-Phytate + blue dye (in only four patients)	10: normal ovarian cortex 25: proper ovarian and suspensory ligament	10 min	Aortic only 84%/ pelvic only 8%/ both aortic and pelvic 8%	Cortex injection: 40%/0% ligaments injection: 84%/0% radiotracer 71.4%/0%
Angelucci/2016 [18]	Early ovarian carcinoma/5	ICG	Hilum of the ovary	2 min	Aortic only 40%/ pelvic only 20%/ both aortic and pelvic 40%	100%/NA
Buda/2017 [19]	Suspicion of malignant ovarian tumor (7 patients) + cervical carcinoma (3 patients)/10	ICG	Dorsal and ventral side of the proper ovarian and suspensory ligament	Real time	Aortic only 67%/pelvic only 11%/both aortic and pelvic 22%	90%/NA
Speth/2017 [20]	Three endometrial cancer G3/3 ^*∗*^	Tc-99m—albumin nanocolloid + blue dye	Proper ovarian and suspensory ligament	15 min	Aortic only 67%/pelvic only 33%	100%/NA
Nyberg/2017 [21]	Ovarian mass (cancer = 5, benign = 11, borderline = 4 patients)/20	Tc-99m—albumin nanocolloid + blue dye	Mesovarium	10–20 min	Aortic only 60%/pelvic only 10%/both aortic and pelvic 30%	100%/0%
Lago/2019 [12]	Early ovarian cancer/10	Tc-99m—albumin colloid +IGC	Proper ovarian and suspensory ligament stumps	15–30 min	NA	Tc-99m:100% (IGC: 90%)/50%
Uccella/2019 [13]	Early ovarian cancer/31	ICG	Dorsal and ventral side of the proper ovarian and suspensory ligament	5–20 min	Aortic only 62%/ pelvic only 19%/both aortic and pelvic 19%	67.7%/0%
Lago/2020 [22]	Early ovarian cancer/20	Tc-99m—albumin colloid + IGC	Proper ovarian and suspensory ligament stumps	15–30 min	Aortic only 5%/ both aortic and pelvic 95%	Tc-99m:100%/NA IGC: 95%/NA
Laven/2020 [23]	Pelvic mass suspicious for malignancy (8 patients) or with a history of prior resection of a malignant ovarian mass (3 patients)/11	Tc-99m—albumin nanocolloid + blue dye	Dorsal and ventral sides of the remains of the proper ovarian and suspensory ligaments	At least 15 min	Aortic only 18%/ both aortic and pelvic 9%	Tc-99m: 27%/NA blue dye: 0%/NA
The current study	Suspicion of malignant ovarian tumor/30	Tc-99m-phytate	Proper ovarian and suspensory ligament	15–20 min	Aortic only 20%/pelvic only 23%/both aortic and pelvic 47%	90%/NA

^*∗*^Eight patients were considered in this study. Of these, five cases with an ovarian tumor were published elsewhere [20]. As such, these five patients were excluded from the study in question. ICG, indocyanine green; Tc-99m, technetium 99; NA, not available; SPECT/CT, single-photon emission computed tomography/computed tomography.

## Data Availability

The data used to support the findings of this study are available from the corresponding author upon request.
